# Massive-Scale Data Mining to Enhance Digital Library with Applications in College Education

This article has been retracted.

**DOI:** 10.1155/2022/9698477

**Published:** 2022-06-16

**Authors:** Chunyan Xu, Jing Bai

**Affiliations:** Zhengzhou Preschool Education College, Zhengzhou 450000, China

## Abstract

The context of digital library has changed from insufficient information to information overload, and its corresponding service mode should also change from “people looking for information” to “information looking for people.” Using a grounded theory approach, this paper extracts 78 initial concepts, 24 basic categories, and 6 main categories by coding and analyzing the raw data obtained from the interviews. On this basis, the relationship path and action mechanism between categories are discovered; based on which a theoretical model of the influence mechanism of digital library intelligent information recommendation service satisfaction is constructed. The research results have shown that, under the moderating effect of user preference, the quality of data mining system, recommendation information quality, recommendation service quality, and recommendation form together have an impact on the satisfaction of digital library intelligent information recommendation service. The results of our work can provide useful reference for the optimization and healthy development of digital library services. Meanwhile, it has some theoretical and practical contributions. How to quickly obtain the information people required from a large amount of information is particularly important. Personalized construction is an inevitable service trend for the development of digital libraries in the new era. We in this paper study the current situation of digital libraries and the development of personalized services in digital libraries. We focus on data mining-related technologies, the development of digital library data exploration technologies, and the provision of Internet application services. The problems in this area were summarized, and the countermeasures were put forward based on this. It can be concluded that the concept of a digital library is not just a collection of data with information management tools, it is an environment that brings together collections, services, and people to support the entire data flow. It converts information into domain knowledge, from creation to dissemination. It guides the process from use to save. The trial registration number is ChiCTR2200055403.

## 1. Introduction

With the development of enlightenment technology, on the one hand, rich information content satisfies the life of modern people; on the other hand, a large number of people acquire knowledge by using the Internet, that is, using the digital libraries. With the increase of digital library users, people's requirements for the personalized benefits of digital library are also getting higher and higher. In order to obtain the information you do not acquire from the massive information, data mining technology is pervasively used nowadays. The application of uncertainty deep data mining technology in digital library can improve the screening efficiency of narrative list information in digital library. It can enrich the personalized services on the basis of digital libraries. Also, it can improve the needs of added digital library users for information recovery and account book versions. Further, digital libraries will be hurt due to users' reading habits [1].

Prescribing individualized utilization methods for users has become an indispensable primary problem for every digital library administrator. It is also an important way to interpret products in a way similar to web advertising. The University of Michigan proposed the establishment of an electronic library in 1990 and established a popular standard set by the miscellaneous department privately associated with reading rooms. The holdings standard was identified as a digital library. This article does not consider the test division of the digital library and does not elaborate too much on this point. It is specifically explained as a software system that uses the expression of numbers and several technical skeletons to restore various information in it [2]. Data mining recommends using market evaluations to consume the size of cryptic information from data, extracting and supporting data rules by removing and referencing uncertain knowledge, using statistics, retrieval notification databases, and diverse fork identification to check what is available in the database. Data is emerged for data management and usage rules; it is possible to enter precise nouns to mine problems and mine information for control [3]. The key techniques of cunning data mining are bundle method, taxonomy and divination method, joint method, and offensive discovery method. The frequently used models are decision trees, backtracking analysis, cunning neural networks, etc. To build a digital library, only when the above technologies are fully connected can a digital library with its own characteristics be built well.

The example of the personalized system of digital library should be user-centered and focuses on the operability, constructiveness, and renewability of digital library. It should dismantle and mine users and book funds. The design of data mining personalized digital library system example is to mine digital library users' personal instructions and online behaviors and analyze users' hobbies, literary works, and etiquette habits. The objective is to provide users with high-quality celebrities. It provides the basis for the vestibule of library rules [4]. We analyze and design, disassemble user behavior, perform cluster analysis based on user registration notices, extract, browse, reflect, classify, and provide different service methods and evaluation methods for different nests. Meanwhile, books with a large number of lists have a large audience and should be shared. The login close page or locate in the citations section is designed for the library's general ledger. The system establishes a user model coordinated with the user's registration and login information in the digital library. An information database management system is coordinated with the user's recovery records. The system matches user solutions with intelligent bases and provides users with personalized intelligent services through twinning problems. According to the user's registration prompt, recycling information, and course selection information, we establish a user information database and an information fund database. The personalized system will call the user means library and information resource library, sort the users and establish the use rights and responsibilities model, and use data mining technology to find users. Interested in funding, we propose the so-called recommend users. The personalized service of the digital library is that the digital library provides customized services for different users in different places and residences. Mainly in the user's personalized information customization and notification embarrassing service, the user's registration suggestion and envelope record burst bearing are leveraged to formulate the user's necessary database management system. These results are subsequently fused by the system uses data mining technology and other information technology to mine users. We follow the information and send it to the user. According to the purpose of the updateability of the digital library, the system will update the user's real-time personal database in the future work to meet the user's real-time information procurement needs.

## 2. Related Work

Digital libraries have foreseen the academic resorts that users can choose [1–10], but with the explosive effect of academic resources, the phenomenon of digital library information overload has become more and more serious [11], and finding a suitable academic resort has become a huge problem [11, 12] and using recommender system support to address this problem [13]. With the help of the recommendation system, the relevant intelligence is “pushed” to the digital library users so that they can keep more benefit [10]. Therefore, it is involuntary for digital libraries to interest recommender systems as a singular drive to forward and speed up ailment examine tenon [14]. Recommender systems, also known as personalized recommender systems [15], can pressingly satisfy personalized science and foresee peculiar learned mean to verify usage activities [12]. Proper use of recommender systems is not only critical to provide a truly personalized office but also helps reduce information overload and improve user exercise satisfaction [14]. Recommender systems have been regarded as an important research site since the timely 1990s [16]. In 1992, the Xerox Institute in the United States improved the Tapestry system [17] program to filter compressed e-mails and recommend electronic gossip, an old way for commercial organizations to recommend information resources. In the mid-1990s, the requirements of recommender systems were extended to answers for digital libraries, and the American libraries diligently pioneered the purpose of developing recommender systems for digital libraries. In 1995, Balabanović and Shoham of Stanford University proposed the purpose of their beloved recommender system for digital libraries and launched a part of jut, the personalized evaluation system LIRA [18]; in 1997, they initiated the project's another shot. The first is the personalized recommendation system Fab [19]. In 1998, Bollacker et al. [20] proposed the academician resource respect system CiteSeer, which attracts the attention of the community from all aspects of life. In the same year, the American Association for Artificial Intelligence (AAAI) organized a special conference to focus on the development of recommender systems [15]. Around 2000, Cornell University Library took the lead in breaking through the relatively mature library personalized office system My Library@Cornell system and provided a purpose model for many subsequent digital library witness systems [11]. Since then, the personalized witness utility of the digital library has gradually improved. However, in recent ALICE, the imposition of platonic designs by users has shown an open tailing trend [12], which places higher demands on the suggestion system. In the past, the product of the conspiracy of recommendation systems and modern information technology perceived recommendation came into being. The application of understanding respect in the field of notification resources is intelligent information proof, that is, computer information systems actively provide users with information that matches their interests, preferences, or indispensable by decomposing user data, order notification.

Intelligent murmuring testimonial is an essential part of the personalized benefit of digital library. As cultivated news doorkeeper in an unworn era of revelation, scholars from omen and incorrect have grown more and more excited near the investigation on communicative complaint testimonial for digital libraries. At present, the research on intelligent recommendation of the Texas Digital Library mainly focuses on algorithm and technology, system and model, cosecant and utility, etc. In algorithmic rules and technologies for intelligent information recommendation in digital libraries, Guo et al. [9] provide personalized proof orders for digital resources, integrating PageRank and Collaborative Filtering (CF) technologies into a unified framework, a time-aware network that generates and dissects user and resort relationships from historical usage data. Appropriate digital resources are submitted to active digital library users. For the proposed system and standard for intelligent guidance of digital library, Tian et al. [14] proposed a personalized evaluation system for institutional libraries based on mixed proof algorithm program support, which allows users to select an appropriate ledger from among many trial accounts. On the role and benefits of understanding prompt recommendations in digital libraries, Li He et al. [16] found that, as a new type of mobile library information service, the situation-aware teaching witness office has a marked personalization advantage, and the matching of technology and equipment is the most important factor in this service. The service anticipates external motivations and important assurances. As research matures, more and more proficient information proof systems are used or become the touchstone of digital libraries, such as proficient book recommendation systems [15], scientific research paper recommendation systems [16], biomedical journal compliance recommendation systems [7], inspector testimonial system [8], and skilled reserve {2} auxiliary display quotation system [16]. The practice of intelligent information recommendation in digital libraries is being further deepened.

To sum up, the major exploration has carried out the necessary activities, but there are still occupational deficiencies. The research on smart advertising certificates in existing digital libraries mainly focuses on the frontend of the understanding of smart certificates, that is, taking the necessary use as the next step, vigorously dispersing the export of “how to network” and “how to optimize” in terms of technology, algorithm programs, models, etc. However, few statement meditations concentrate on the back limit of intelligent sorrow advice, that is, starting from the unavoidable necessity, considering the test of “what to execute” and “what to optimize” in stipulation of testimonial temper and recommendation performance. However, from the appearance of user having contentment, the retrospect of digital library cognitive disorder testimonium service is even rarer. Secondly, the existent examination of the contentment with the manner of digital libraries has greatly dispersed the bandage force or appraisement indicators for user indemnification [18–20], while the digital library actually provides many useful things, such as seat-only books, borrowing and returning books, advertising, and consult. There may be differences in different specific purpose strike devices, and more in-depth targeted research is required to experience it.

## 3. Our Proposed Method

In the pipeline of our digital library system, all notification summaries of information storage are stored in the database server. Thus, the version instructions of data information do not need to be transmitted through the network. This relies on intelligence classification to simplify the intelligence mining procedure, overcome reticulum detention, and avoid running plans. We attempt to reduce the data weight of the network and program-based modularization. This can design a stable storage process. After the first data storage is completed, the subsequent similar transaction operations can follow the first factory tautology. If the notification of storage occurs, then the database tray will constitute an embarrassment suitable for education. The notification storage protrusion of the system is shown in Figure 1. In this system, the program list summaries stored in the message are all stored in the database management system server. Therefore, there is no need for reading instructions for data advertisements. It must be transmitted through the network, which depends on the intelligent classification to simplify the information mining process, reducing grid delay. This avoids the factory thrust and reduces the weight of mesh data. Subsequently, the specific operations can be repeated. We agree to the first notification if the stored notifications are diversified. Besides, a similar advisor will be constituted in the database salver and information storage process to block the system as shown in Figure 1.

The interpretation saver of the decision tree algorithm rules is to discover valuable advertisements from all the personalized interactive service messages certified by the system. We further classify them in detail and in the partition tree constructed by the system. One node corresponds to an honest attribution, as one of this standard. The output event is represented by a branch. Assuming that node *R* is the complaint rule applying for accumulating class *C*, the system will automatically select the attribute with the highest elegant rate to burst it. In this dilemma, celebrities are similar to interactive puzzle judgments for thinking enlightenment. It can be expressed as formula (1). Pz is the probability that the fixed tip in the message clot represented by *C* can be refined into a G-type tip. After the system completes the recommended polishing and classification, it can be estimated by

(1) $$\begin{array}{c} \text{dist}=\left|C-d\;\right|\left./\right|\;D, \end{array}$$

where *C* represents the badness of *C*. If attribute *A* of the personalized interactive service information can be represented by several different values, then the enlightenment prompt with the characteristic *A* in the C-type enlightenment rules corresponds to the request information which can be expressed as

(2) $$\begin{array}{c} \text{InfA}\left(C\right)=H\left(x\right)\log T+\text{Info}\left(G\right). \end{array}$$

In this formula, InfA(*C*) is the advertisement obtained after classification of *C* information embarrass corresponding to attribute *A*, the system will automatically adopt the minimum trust notification reciprocal attribute to consider splitting *c*.

In this paper, the semistructured meeting method is used for data stacking, and the data collection progress is shown in Figure 2. Through literature survey and previous contacts, a preliminary interview outline was designed, two interviewees were called for prequestioning and revision, and the formal meeting outline was firm. In the interview sketch, the embarrassing four aspects are introduction, word definition, interviewee's suggestion, and core question. In this paper, samples are selected according to the principles of purposeful attempts [6] and theoretical saturation attempts [7]. From the beginning of the whetstone specimen, this concern describes the eligibility of the specimen's appearance as follows: (1) a digital library that is domestically owned and regularly worn; (2) it has contacts or is respected by the office for sensitive information; (3) it can clearly interpret interview questions and has the ability to clearly express one's own knowledge, opinions, and ideas; (4) it has the ability to specify the maximum amount of information for doubtful points of the question.

According to the principle of theoretical saturation sampling, close the digital library before the respondent no longer provides novel categories. We prove it with more than 3 people and a postbending study sample. Combined with the above ethical norms, we in this paper argue that graduate student gatherings with educational frankness and violence are digitally native gatherings (innate in 1990 and later). Their feelings about the near-cognitive advertising witness benefits of digital libraries are more typical. Huge research is based on sampling the docking family. At the same time, it is convenient to get enough tips to achieve doctrinal purity by communicating with teachers and students who need digital libraries more frequently. At the same time, taking into account the convenience of data collection and taking account of narrative alternatives such as different genders and different majors as much as possible, this newspaper finally selected 21 respondents as the test subjects.

The data acquisition performance of this article is approximately 9 weeks. At the composing question level, data compilation is implicit through online interviews. Meanwhile, interviews are recorded with the user's permission. During interviews, interviewees were asked almost anything that was unclear or ambiguous. After the interview is over, it will be copied through data processing software and manually proofread and revised. After this, it is sent to the respondents for verification to ensure the authenticity of the data and is represented by symbols A to U in the order confirmed by the respondents.

## 4. Experimental Results and Analysis

The presentation is three-dimensional, heterogeneous, functional, and factual, with mandatory project interactivity and effective sketch extensibility. The combination of reality and technology satisfies the librarian's creative understanding of the peculiar library. The combination of pinna, visual, and tactile judgments, coinciding with a more active three-dimensional digital library, is an elite medium for drone education and library limelight. Combined with the new library system and rational development in three-dimensional space, library services will be more personalized and humanized. The creative expansion of the library's digital resort has revolutionized the use of library expedients. Functional structure: navigation—book search navigation: system navigation cosine: users can click on the retrieved books to navigate the books they are interested in. The system will automatically calculate the best path and present it to the user in the form of screenshots and 3D navigation techniques, and will guide the use to the situation where the leger is restored. Interaction—personal center: personal center: users can create their own nickname and chattel sketch in the wares correctness center. Then, disclose the usage of actually active in participation vitality activities, interacting with other readers in the community, chatter with other readers, atmospheric and using reading lodge, fire training and escapes and a series of hands-on activities. Interact—chat with friends. Make boyfriend chat: find and cosponsor through account and name, conduct interactive online communication, and increase the fun. Interactive—virtual consultation: virtual consulting slavish forms a consultation desk on the virtual floor and brings together avatars. Readers can contact a counselor with questions about the library. Some results are shown in Figure 3.

Fact advisors can ask the usual consulting questions, or library sponsors can rebut points online. For the schematic diagram of the functional structure, see Table 1. Virtual showroom—movie screening room: the picture screening room is a potential screening seat in the library. Students can select their own films for screening, and the library can also upload videos of student activities to the screening room. Libraries can also set up an ethics webinar vestibule with videos condemned by experts and scholars. Virtual retirement house—an extraordinary collection of experienced monographs: the library's own precious and outdated monographs can be expanded on a three-dimensional moral highway and made available to students for reference. Virtual showroom—database showroom: when delivered, each library purchased a dozen or even hundreds of database resources, but most libraries were embarrassed that the database usage rate was not violent. Libraries are looking for ways to promote databases to inspire readers' knowledge. In order to make readers like to look at the database and understand the database, the 3D physical digital library deliberately displays the database on the potential floor, virtualizing the electronic funds as an “external” library collection resort. Diversify the library's existing database to each performance entry through expert classification such as paper recycling front office, industry announcement hall, e-library hall, video lecture front office, and concord hall. Then, in each showroom, there are profiles and links to relevant databases to speak. Readers can wander through the various galleries, agreeing on their interests and indispensability. The underlying “physical” formulation of this electronic means can allow readers to more intuitively and trivially test the creatures of electronic resources and curiously own and learn about them. Second, the number of databases is relatively complete, which is convenient for readers to cite. By placing similar lined databases in the exhibition hall, it is convenient for readers to compare and use, and readers' feedback on the data obtained by the library can be predicted in advance. Interactive game—doodle painting: students can engage in doodle art and upload their duties. Through the voting and scoring system, excellent works are selected and displayed on the cave painting column for everyone to appreciate and increase interactivity. The system can also adjust and upload other literati emblem entries. Interactive front hall: 3D psychedelic games can be loaded, allowing students to embellish knowledge in entertainment. Interactive project—comparison front office: the practical comparison hall adopts the technology of stimulating individuality and multiperson online, which can be used for librarians to continue to hold meetings, student associations to hold meetings, etc. Before the intersection, there is a room for the library of the practice meeting.

Our library lecterns are designed to be easy to use and flexibly adapt to each librarian's own library. The platform is highly open, from the choice of building type to every facility in the country which can be tailored according to needs. The platform showcases the difference in size, and readers can upload their own descriptions, sound, and video expedients to the resort library depending on the format, which then unfolds creatively in three-dimensional time. Readers specify their own fact base, which can be saved and uploaded to the assigned course, and excellent works are selected through the scoring system for other readers to edit. Functions: (1) readers can deepen their understanding of the library by building their own practical library. By arranging their own virtual tours, readers can show off their creativity and grace and enjoy the physical earth. Libraries can let students participate in the arrangement through competitions, guide readers' activities, and demonstrate teacher training and effectiveness. Through the Build My Library movement, the library supports the concept of a virtual library so that students will want and learn to customize a physical library. System framework performance module—basic construction: the basic production of my library on the 2D page, including the quotation and construction of library types, doors, windows, floors, and layout, as well as the interior layout of indoor hardware facilities, and the basic construction structure through the 2D account plan. Afterwards, you can point to 3D pages, foresee construction signs, and make listless adjustments to the location of indoor facilities. Function module—content: select the description text, audio and video, and text and other content in the material library on the right, and creatively add it to the 3D exhibition as a hotspot or image source. Functional model—3D rove: click on the rove cosecant to roam through the de facto time already formed and decorated. With video recording, you can record the scope process through command events and save or upload your own recordings. Functional module—my study room: my study room can accumulate your number one account book; you can access pericope's account book database via hyperlink; you can schedule your own reading practice, write yourself a story, and read a book with everyone book [20, 21].

## 5. Conclusions

Under the tide of informatization, digital library will be presented in front of the world with a new look and provide the public with knowledge services anytime, anywhere. This requires builders to have a clear understanding of the digital wave in the information age, not only to see the convenience brought by digitalization but also to see the challenges that digitalization brings to existing businesses. In order to solve the problems of slow response and poor sharing of the traditional digital library interactive service system, this paper designs a digital library personalized information interactive service system based on digital mining technology and introduces the improved design based on the traditional system. The new system architecture expounds the controller design with TQMA93RE7 ultra-high-density chip as the core and the information storage process design of the modular program and explains the construction basis and method of the decision tree algorithm. The comparative test results of the system show that the average time and information of this system are comparable to other systems, which can greatly improve the user experience of library users.

## Figures and Tables

**Figure 1:** An example of the storage protrusion.

**Figure 2:** An overview of our designed data mining-based digital library framework.

**Figure 3:** Response time comparison under multiple attributes.

**Table 1:** System stability evaluation.

Concurrency level	Textual system		System [6]	
	CPU usage	Ram usage	CPU usage	Ram usage
500	34%	27%	41%	35%
1000	41%	32%	47%	38%
2000	40%	44%	48%	49%
3000	32%	32%	39%	41%
4000	55%	34%	61%	40%

## Data Availability

The data used to support the findings of this study are available from the corresponding author upon request.
